This article has been retracted.

# Aerobic Degradation of *N*-Methyl-4-Nitroaniline (MNA) by *Pseudomonas* sp. Strain FK357 Isolated from Soil

**DOI:** 10.1371/journal.pone.0075046

**Published:** 2013-10-08

**Authors:** Fazlurrahman Khan, Bhawna Vyas, Deepika Pal, Swaranjit Singh Cameotra

**Affiliations:** Environmental Biotechnology and Microbial Biochemistry Laboratory, Institute of Microbial Technology, Council of Scientific and Industrial Research (CSIR), Sector 39-A, Chandigarh, India; Centro Nacional de Biotecnologia - CSIC, Spain

## Abstract

*N*-Methyl-4-nitroaniline (MNA) is used as an additive to lower the melting temperature of energetic materials in the synthesis of insensitive explosives. Although the biotransformation of MNA under anaerobic condition has been reported, its aerobic microbial degradation has not been documented yet. A soil microcosms study showed the efficient aerobic degradation of MNA by the inhabitant soil microorganisms. An aerobic bacterium, *Pseudomonas* sp. strain FK357, able to utilize MNA as the sole carbon, nitrogen, and energy source, was isolated from soil microcosms. HPLC and GC-MS analysis of the samples obtained from growth and resting cell studies showed the formation of 4-nitroaniline (4-NA), 4-aminophenol (4-AP), and 1, 2, 4-benzenetriol (BT) as major metabolic intermediates in the MNA degradation pathway. Enzymatic assay carried out on cell-free lysates of MNA grown cells confirmed *N-*demethylation reaction is the first step of MNA degradation with the formation of 4-NA and formaldehyde products. Flavin-dependent transformation of 4-NA to 4-AP in cell extracts demonstrated that the second step of MNA degradation is a monooxygenation. Furthermore, conversion of 4-AP to BT by MNA grown cells indicates the involvement of oxidative deamination (release of NH_2_ substituent) reaction in third step of MNA degradation. Subsequent degradation of BT occurs by the action of benzenetriol 1, 2-dioxygenase as reported for the degradation of 4-nitrophenol. This is the first report on aerobic degradation of MNA by a single bacterium along with elucidation of metabolic pathway.

## Introduction

*N*-Methyl-4-nitroaniline (C_7_H_8_N_2_O_2_, MNA) is a nitroaromatic compound, used as an additive for lowering the melting temperature of highly energetic compounds, such as 2, 4-dinitroanisole (DNAN), that helps in easier synthesis of insensitive explosives [1], [2], [3]. During the process of manufacturing, packaging, and handling of insensitive explosives, it may get released into the environment through various waste streams [2]. Presence of electron withdrawing nitro group (−NO_2_) in the benzene ring results in acute toxicity to human and other life forms [2], [4]. As a result of toxicity and recalcitrant nature of nitroaromatic compounds, public concern has prompted the need to develop clean-up technologies for restoration of environments. Microbial degradation/or transformation could be used as an effective mechanism for the elimination of nitroaromatic compounds from the environment. Microbial degradation of nitroaromatic compounds can take place in both aerobic and anaerobic conditions, however, due to electron withdrawing effect of nitro group, only nitro group is reduced sequentially into aryl nitroso (Ar-NO), aryl hydroxylamine (Ar-NHOH), and aryl amine (Ar-NH_2_) without any aromatic ring cleavage [5], [6]. These reductive transformations have been shown to be slow and the reductively transformed products are known to be carcinogenic [7], [8], [9]. The oxidative degradation of recalcitrant compounds under aerobic conditions is expected to be one of the most effective mechanisms for rapid and complete mineralization, which occurs by non-specific enzymes [10], [11], [12]. There are few reports on biological transformation of MNA in anaerobic fluidized-bed bioreactors, where MNA was reductively transformed into 4-methoxy-phenylenediamine that gets accumulated as dead end product followed by dimer formation [1], [2]. Till date there is no information available on aerobic transformation/or degradation of MNA by means of bacterial isolates. Elucidation of catabolic pathways involved in degradation of xenobiotic compounds is critical for both ‘basic understanding’ and ‘development of remediation technologies’ [13], [14], [15]. Therefore, studies on isolation of MNA degrading aerobic bacteria and elucidation of corresponding metabolic pathways are of great ecological significance. In this communication we report isolation of a bacterial strain *Pseudomonas* sp. strain FK357, isolated from soil that utilizes MNA as the sole source of carbon, nitrogen, and energy. The degradation of MNA by strain FK357 occurs via the formation of 4-NA, 4-AP, and BT as the major metabolic intermediates. We propose that strain FK357 could be used as a model system for studying the molecular and biochemical mechanism of aerobic degradation of MNA as well as for the development of MNA bioremediation technology.

## Materials and Methods

### Chemicals and Growth Media

*N*-Methyl-4-nitroaniline (MNA), 4-nitroaniline (4-NA), 4-aminophenol (4-AP), and benzenetriol (BT) were purchased from Sigma-Aldrich (St, Louis, MO, USA). Minimal salt medium (MSM) used in the present study was prepared as described earlier [16] with slight modification i.e. absence of nitrogen source [(NH_4_)_2_SO_4_]. Stock solution (10 mM) of MNA prepared in HPLC grade methanol was added to an empty Erlenmeyer flask to obtain the working concentrations. Further, the residual methanol in the flask was evaporated under stream of air to leave the dry crystal of MNA in the bottom of flask. Nutrient agar (NA) and nutrient broth (NB) both at one-quarter strength (1/4^th^) were used as rich media for bacterial growth and culture maintenance.

### Soil Microcosms Study

The non-polluted soil sample was collected from the lawn of Institute of Microbial Technology, Chandigarh, India. The pH of the soil was 5.9, and it consisted of 8.2% moisture, 3. 5% total organic carbon and 1.7% total nitrogen content, respectively. The soil samples were sieved through 2 mm mess to remove stones and debris. Soil microcosms experiment was carried out as described previously with slight modification [17]. Subsequently, 5 gm soil sample was suspended in 50 ml MSM in 250 ml Erlenmeyer flask supplemented with 100 µM MNA. Further, the above microcosms were each supplemented with or without (i) 10 mM glucose and 5 mM succinate as the sole carbon source, or (ii) 0.8 g L^−1^ NH_4_Cl as the sole nitrogen source, or (iii) 10 mM glucose, 5 mM succinate and 0.8 g L^−1^ NH_4_Cl as the sole carbon and nitrogen source, respectively. A control was also set up containing 5 gm autoclaved soil in 50 ml MSM and MNA (100 µM). All the above flasks were incubated in dark at 30°C under shaking condition (150 rpm). At regular time intervals, samples were withdrawn from the test and control flasks and analyzed for the disappearance of MNA. All the experiments were carried out in triplicates.

### Isolation and Characterization of MNA Degrading Bacteria

Upon complete depletion of MNA in the soil microcosms, the serially diluted soil slurries was spread plated on selective medium (MSM-agar containing 700 µM MNA) and incubated at 30°C for one week. The bacterial colonies appeared on the plate were selected for characterization and were tested for MNA degradation. The selected bacterial isolates were used for primary screening by inoculating in 10 ml vials containing 3 ml carbon-free MSM supplemented with different concentrations (50–700 µM) of MNA. The positive bacterial isolates were selected on the basis of increase in growth accompanied by substrate depletion and release of ammonia (NH_4_^+^) and nitrite (NO_2_^−^) ions as measured colorimetrically at wavelength of 340 and 540 nm, respectively. Purity of the positive isolates was checked by streaking on 1/4-NA plates. Further, the efficient MNA degrading isolate was identified using polyphasic taxonomy and 16S rRNA gene sequencing [17]. The 16S rRNA gene sequence (1431 base pairs) of strain FK357 was compared to those of the type strains of *Pseudomonas* using the BLAST search.

### Growth Studies and Degradation of MNA by Strain FK357

The growth studies of strain FK357 and degradation of MNA were performed in 50 ml carbon-free MSM supplemented with varying concentrations of MNA ranging from 50 to 700 µM by inoculating (1%, v/v) seed culture grown in 1/4-NB. The flasks were incubated at 30°C under shaking condition of 200 rpm. At every 8 hours, culture was withdrawn and optical cell density at 600 nm (OD_600_ nm) was measured using Lambda EZ 201 UV-visible spectrophotometer (Perkin-Elmer Inc, USA). The bacterial growth was also monitored by measuring the total protein of the culture with the help of Pierce BCA protein assay kit (Thermo Scientific, USA). Culture fluid samples (2.0 ml) were centrifuged at 8,000 × g for 10 min to obtain cell-free supernatants which were used for analysis of the amount of NH_4_^+^ and NO_2_^−^ released. Subsequently, the above supernatants were also used for the quantitative determination of MNA disappearance and identification of metabolic intermediates by HPLC. Non-inoculated and inoculated flasks with heat killed cells of strain FK357 were used as abiotic and negative controls, respectively. Another control experiment was also conducted by inoculating strain FK357 in carbon-free MSM (not supplemented with MNA).

### Resting Cell Studies

Resting cell studies on MNA degradation were carried out according to the method described elsewhere [18]. The overnight 1/4-NB grown seed culture (6%, v/v) of strain FK357 was inoculated into 1.0 L of 1/4-NB supplemented with MNA (150 µM) and incubated at 30°C under shaking at 200 rpm up to 24 hours. Similarly, to obtain un-induced cells, the strain FK357 was grown in 1/4-NB only. When the optical cell density of the culture reached to OD_600_ ranged between 1.2–1.5, the cells (induced and un-induced) were harvested by centrifugation at 8,000×g at 4°C for 10 min, washed twice with phosphate buffer (20 mM, pH 7.2) and suspended in 100 ml carbon-free MSM. In 25 ml cell suspension 150 µM each of MNA and 4-NA were supplemented separately. Similarly, the degradation of MNA and 4-NA by un-induced cells were also carried out by suspending the un-induced cells in 25 ml MSM supplemented with 150 µM each of MNA and 4-NA, separately. Non-inoculated and inoculated flasks with heat killed cells were used as abiotic and negative controls, respectively. Each flask was incubated at 30°C with shaking at 150 rpm. Samples (2.0 ml) were withdrawn from both control and experimental flasks at regular time intervals of 2 hours and were analyzed for the amount of NO_2_^−^, and NH_4_^+^ released, followed by High Performance Liquid Chromatography (HPLC) and Gas-Chromatography Mass-Spectroscopy (GC-MS) analysis (methods described later).

### Enzyme Assays with Cell-free Lysates

MNA-induced cells of strain FK357 were harvested by centrifugation and washed twice with phosphate buffer (20 mM, pH 7.2) and re-suspended in phosphate buffer. The cell suspensions lysed by passages through a French pressure cell (20,000 lb/in^2^) were centrifuged at 12,000 rpm for 30 min at 4°C and supernatant was separated to obtain cell-free enzyme extract, which was subsequently used for the enzyme assays. Protein content within cell-free extracts was determined with Pierce BCA protein assay kit (Thermo Scientific, USA). The cell-free extract was used for determining activities of *N*-demethylase, monooxygenase, and 1, 2, 4-benzenetriol 1, 2-dioxygenase, respectively as described below.

#### Enzyme assay for *N*-demethylase

Demethylation reaction i.e. removal of *N*-methyl group from MNA in cell-free lysates was carried out according to the method of Summers et al. [19]. The reaction was carried out in a total volume of 10 ml phosphate buffer (50 mM, pH 7.5) containing cell-free protein (2.0 mg ml^−1^) 150 µM NADH, 25 mM Fe (NH_4_)_2_(SO_4_)_2_·6 H_2_O and 150 µM MNA. The enzymatic reaction was initiated by addition of 150 µM MNA and incubated at 30°C under shaking (200 rpm). The control reactions lacking either substrate or cell-free protein were also used during the above reaction. The *N*-demethylase activity was determined by measuring time dependent depletion of substrate and formation of *N*-demethylated product by HPLC. The formation of formaldehyde (HCHO) in the demethylation reaction was quantitatively determined by using an assay based on the Hantzsch reaction [20]. Briefly, in 0.5 ml of culture supernatant equal volume of reagent B (2 M ammonium acetate, 0.05 M acetic acid and 0.02 M acetylacetone) was added and incubated at 58°C for 5 min. Presence of HCHO in the sample was determined colorimetrically by calculating the absorbance at 412 nm as the HCHO adduct diacetyldihydrolutidine.

#### Enzyme assay for monooxygenase

The monooxygenase mediated conversion of 4-NA into 4-AP was carried out in cell-free lysates prepared from MNA grown cells of strain FK357 as described previously [21]. The reaction was carried out in a total volume of 10 ml phosphate buffer (20 mM, pH 7.0) containing cell-free protein (2.0 mg ml^−1^) 200 µM NADPH, 150 µM FMN. The reaction was initiated by addition of 100 µM 4-NA and incubated at 28°C. The control reactions lacking either substrate or cell-free protein or cofactors (NADPH or FMN) were also used during the above reaction. The monooxygenase activity was determined by measuring time dependent depletion of substrate and formation of product by HPLC. Similarly, quantitative determination of NO_2_^−^ ions released in the above reaction was also estimated colorimetrically.

#### Aniline dioxygenase assay

The dioxygenation reaction involved in the conversion of 4-AP to BT by strain FK357 was measured with an oxygen electrode (YSI, Ohio, USA), according to the method as described previously [22], [23]. MNA-induced and un-induced cells (as described in the resting cell study) were harvested by centrifugation at 7,500×g at 4°C for 15 min. Pellets were washed twice with phosphate buffer (20 mM, pH 7.2) and re-suspended in the same buffer. This suspension was used for the assay of dioxygenase by measuring oxygen uptake at 30°C. The reaction was carried out in 1.85 ml volume air-saturated phosphate buffer (20 mM, pH 7.2) containing substrates (70 µM), and cells (0.25 mg of protein).

#### 1, 2, 4-Benzenetriol 1, 2-dioxygenase enzyme assay

It is known that the degradation of terminal intermediate 1, 2, 4-benzenetriol (BT) starts by the action of 1, 2, 4-benzenetriol 1, 2-dioxygenase with the formation of lower pathway intermediate i.e. maleylacetate (MA) [24]. 1, 2, 4-Benzenetriol 1, 2-dioxygenase activity was determined spectrophotometrically using Lambda EZ 201 UV-visible spectrophotometer (Perkin-Elmer Inc, Massachusetts, USA) [21]. The reaction mixture consisted of 50 mM sodium phosphate buffer (pH 7.0), 10 mM Fe (NH_4_)_2_(SO_4_)_2_·6 H_2_O, and 0.5 mg soluble protein of cell-free lysates, in the total reaction volume of 1.0 ml. Reaction was initiated by the addition of 70 µM of BT to the reaction mixture. Enzyme activity was monitored with wavelength scan over a range of 220–360 nm at an interval of 1 min.

### Analytical Methods

The release of nitrite ions (NO_2_^−^) was monitored with a colorimetric method using N-(1-naphthyl) ethylene-diamine-dihydrochloride and sulfanilic acid reagent as described earlier [25]. The NO_2_^−^ assay was carried out by mixing equal volume (0.1 ml) of reagent A [0.1% (w/v) sulfanilic acid in 30% (v/v) acetic acid] and reagent B [0.1% (w/v) naphthylethylenediamine in 30% acetic acid] to 0.1 ml culture supernatant. Presence of NO_2_^−^ in the sample was indicated by the appearance of purple colour and quantified by calculating the absorbance at 540 nm. Ammonia (NH_4_^+^) concentrations were also monitored with a colorimetric method using ‘Ammonia Estimation Kit’ (Sigma Aldrich, USA) according to the manufacturers’ recommendation. Standard plots generated with known concentrations of (NH_4_)_2_SO_4_ and NaNO_2_ were used to determine the concentrations of NH_4_^+^ and NO_2_^−^ ions. The quantitative determination of MNA and its metabolic intermediates were analyzed by HPLC [21]. The samples collected from growth, resting cell studies and enzyme assays were analyzed by HPLC using Waters-HPLC 2489 model (Waters, USA) equipped with a UV detector and a C-18 reverse phase column at 30°C [21]. The mobile phase used for the separation of substrate and intermediates consisted of acetonitrile: water (30∶70, v/v) under isocratic condition with the flow rate of 1.0 ml min^−1^. The samples were injected with a constant injection volume of 20 µl. The peaks of eluents were monitored with UV detector over a wavelength scan of 220–290 nm. For the GC-MS analysis, samples were prepared by mixing equal volume of ethyl acetate to the cell-free aqueous culture and liquid-liquid extraction performed by layer separation sequentially at neutral and acidic pH. Extracted organic phase was pooled, dried under nitrogen flow using RotaVapor II (BUCHI, Switzerland). The samples were analyzed by GC-MS using QP2010S (Shimadzu Scientific Instruments, USA) as reported earlier [6]. Briefly, the chromatographic separation of substrate and intermediates was carried out with constant temperature of injector, oven, and detector at 280, 200, and 250°C, respectively. Positive molecular ion mass spectra were scanned in mass/charge (m/z) range of 0–160. Identity of different metabolic intermediates was ascertained by comparison of mass fragmentation pattern and subsequent mass spectral database match from the National Institute of Standards and Technology library (NIST).

### Nucleotide Sequence

A total of 1431 base-pairs were sequenced for 16S rRNA gene of strain FK357; which has been deposited to GenBank under the accession no. KF011496.

## Results

### Soil Microcosms Study

The rate of MNA degradation was slightly higher in nitrogen (NH_4_Cl) amended soil microcosms as compared to unamended soil microcosms (Figure 1). The higher rate of MNA degradation in nitrogen-amended soil microcosms, suggests the availability of most favorable nitrogen source from NH_4_Cl, which makes it easier for soil microorganisms to utilize *N*-methyl group as the carbon source. However, in case of soil microcosms amended with a combination of carbon and nitrogen, the rate of MNA degradation was completely inhibited. The inhibition of MNA degradation in the above soil microcosms was likely because the soil inhabitant microorganisms utilized more favorable carbon (succinate and glucose) and nitrogen (NH_4_Cl) source (Figure 1). There was no transformation of MNA in the sterile soil (Figure 1).

**Figure 1:** Biotransformation of MNA in soil microcosms under aerobic conditions. (•), nitrogen-amended; (○), unamended; (▴), carbon-amended; (□), carbon and nitrogen-amended; (▪), sterile. Values are presented as arithmetic mean of data obtained from experiments carried out in triplicate; error bars represent standard deviation.

### Isolation and Characterization of *N*-methyl-4-nitroaniline Degrading Bacteria

After 15 days of incubation, when complete degradation of MNA occurred, the serially diluted soil slurries from microcosms was spread plated on MNA selective plates. Total 35 morphologically different isolates were selected and further screened for the degradation of MNA. Among these isolates, strain FK357 was found to be an efficient MNA degrader. The strain FK357 was selected for the identification and study of MNA degradation along with elucidation of metabolic pathways. Strain FK357 was identified as a facultative anaerobe, Gram-negative, non-spore forming, non-motile, catalase and oxidase positive, rod-shaped bacterium. It showed optimal growth on nutrient rich medium (NA, NB) at 30°C; however it was also able to grow at 37°C. Strain FK357 was found negative for H_2_S production. This strain showed acid production from D-fructose, D-glucose, maltose, D-mannose, D-ribose, trehalose, and L-alanine, whereas, negative on glycerol, D-lactose, D-galactose, D-cellobiose, D-raffinose, and L-serine. Strain FK357 also utilizes acetate and succinate as sole carbon sources. The partial 16S rRNA gene sequence (1431 base pair) of strain FK357 showed 99% sequence similarity to that of several *Pseudomonas putida* strains. Thus, based on the biochemical tests, morphological and physiological characteristics, and phylogenetic analysis, strain FK357 was identified as *Pseudomonas* sp. strain FK357. The strain *Pseudomonas* sp. strain FK357 will be made available to other researchers upon reasonable request.

### Growth Study and Degradation of *N*-methyl-4-nitroaniline by Strain FK357

A growth study of strain FK357 was carried out using different concentrations of MNA ranging from 50 to 700 µM. Growth of strain FK357 was completely abolished at an MNA concentration of 500 µM, whereas 250 µM of MNA was found to be optimal for its growth with subsequent degradation of the parent compound (Figure 2A and B). Strain FK357 grew best on 250 µM concentration of MNA at 30°C and pH 7.2. Degradation of MNA during the growth study occurred with the stoichiometric production of nitrite ions and lesser amount of NH_4_^+^ (Figure 3). The complete depletion of MNA was observed at 96 hours of incubation (Figure 3). Depletion of MNA was accompanied with an increase in growth of strain FK357 as determined by measuring the total cell proteins up to the value of 10.64 µg ml^−1^. A transient accumulation of 4-NA occurred in the media during the degradation of MNA (Figure 3).We were unable to detect formaldehyde (HCHO) during the growth study, while transient accumulation of 4-NA, suggested that the first step of MNA degradation starts via the release of –CH_3_ group in the form of HCHO, followed by the removal of –NO_2_ and –NH_2_ groups, respectively. In growth media the accumulation of released NO_2_^−^ was stoichiometrically up to the value of 249.56±0.17 µM, whereas, a slight accumulation of NH_4_^+^ (51.06 µM) was observed. Thus, non-stoichiometric release of NH_4_^+^ suggested that it might possibly be utilized as a preferential nitrogen source for the growth of strain FK357. The above results are in close agreement with the results reported earlier on the degradation of amino or nitro containing aromatic compounds by different genera of bacteria including *Pseudomonas* [21], [26], [27], [28], [29], [30], [31]. The growth yield of strain FK357 on MNA was found to be 0.55 g of cells/g of MNA. The rate of MNA degradation by strain FK357 was calculated to be 3.26±0.08 nmol MNA min^−1^ mg of protein^−1^. Strain FK357 was unable to grow in MSM in the absence of MNA. The above results indicated that the strain FK357 utilizes MNA as the sole source of carbon, nitrogen, and energy. Growth of strain FK357 on 4-NA was also checked. Strain FK357 also utilizes 4-NA and the degradation of 4-NA occurred via stoichiometric accumulation of NO_2_^−^ and slight accumulation of NH_4_^+^ in the media (data not shown). The growth yield of strain on 4-NA and the rate of 4-NA degradation came out to be 0.43 g of cells/g of 4-NA and 2.73±0.13 nmol 4-NA min^−1^ mg of protein^−1^, respectively. In growth study, we identified only 4-NA as an intermediate; further metabolic intermediates were not identified. Based on the accumulation of NO_2_^−^ and NH_4_^+^ in the growth media, it could be proposed that the subsequent degradation of 4-NA intermediate may initiate either direct ‘oxidative deamination’ of aromatic nucleus or oxidative denitration with the formation of 4-nitrophenol or 4-aminophenol as the putative metabolic product, respectively.

**Figure 2:** Growth characteristics and degradation kinetics of *Pseudomonas* sp. strain FK357 in carbon-free MSM supplemented with different concentrations of MNA. (•), 50 µM; (▴), 150 µM, (Δ), 250 µM; (○), 350 µM; (▪), 500 µM; (□), 700 µM. (A) Growth of strain FK357 on different concentrations of MNA. (B) Degradation of MNA at different concentrations by strain FK357.

**Figure 3:** Growth of *Pseudomonas* sp. strain FK357 on MNA as the sole carbon, nitrogen, and energy source. (•), MNA; (▴), 4-NA; (Δ), NO_2_^−^_;_ (▪), total protein; (○), NH_4_^+^. Values are presented as arithmetic mean of data obtained from experiments carried out in triplicate; error bars represent standard deviation.

### Resting Cell Studies

HPLC analysis of the samples from resting cell study, showed the formation of 4-NA, 4-AP, and BT intermediates as confirmed by comparison with authentic standards. The identified intermediates by HPLC were also confirmed by GC-MS analysis. The mass-fragmentation patterns of the above intermediates viz; 4-NA, 4-AP, and BT were matched with the known authentic standards (Figure 4). Based on the above identified intermediates, we hypothesized that the degradation of MNA occurs via the formation of 4-NA metabolite as a result of demethylation of *N*–CH_3_ group, followed by oxidative removal of –NO_2_ group with the formation of 4-AP. Subsequent degradation of 4-AP may occur by oxidative deamination of –NH_2_ group with the formation of BT as a terminal intermediate.

**Figure 4:** Mass-fragmentation patterns of the metabolites identified by GC-MS analysis during the degradation of MNA by resting cells of *Pseudomonas* sp. strain FK357. (A) Mass-fragmentation patterns of 4-NA (B) Mass-fragmentation patterns of 4-AP, and (C) Mass-fragmentation patterns of BT.

The resting cell study showed that the MNA-induced cells eliminate the lag phase for the depletion of MNA as observed in case of un-induced cells (Figure 5A). Complete degradation of MNA by the induced cells occurred within 6 hours of incubation with the rate of 0.35±0.07 nmol MNA min^−1^ mg of protein^−1^, whereas, un-induced cells degraded MNA after 15 hours of incubation with the rate of 0.17±0.12 nmol MNA min^−1^ mg of protein^−1^. The above results showed that the rate of MNA degradation by induced cells was two times higher compared to the rate of degradation by un-induced cells. The degradation of MNA occurs with the appearance followed by disappearance of 4-NA, 4-AP, and BT intermediates (Figure 5B). The cells pre-exposed with MNA also degraded 4-NA with the formation 4-AP and BT as intermediates and the complete degradation of 4-NA occurred after 10 hours of incubation (data not shown).

**Figure 5:** Kinetics of MNA degradation by MNA-induced and un-induced cells of strain FK357 and identification of MNA degradation intermediates. (A) Kinetics of MNA degradation. (•), MNA; (○), MNA; (▪), MNA in abiotic control. (B) Identification of MNA degradation intermediates. (○), 4-NA; (▴), 4-AP; (Δ), BT. Values are presented as arithmetic mean of data obtained from experiments carried out in triplicate; error bars represent standard deviation.

### *N*-Demethylase Activity (Removal of -CH_3_)

NADH-dependent enzyme assay in the crude cell extract prepared from MNA grown cells catalyzed stoichiometric transformation of MNA to 4-NA (Figure 6A). The conversion of MNA to 4-NA occurred by *N*-demethylation reaction with the removal of –CH_3_ group as determined by stoichiometric formation of HCHO (Figure 6A). The specific activity of *N*-demethylation reaction was found to be 12.33±0.15 nmol min^−1 ^mg of protein^−1^. The identification of 4-NA product from MNA in the enzyme assay confirmed that the first step of MNA degradation is an *N*-demethylation reaction.

**Figure 6:** Stoichiometric *N*-demethylation of MNA and monooxygenation of 4-NA by cell-free lysates prepared from MNA grown cells of strain FK357. (A) *N*-demethylation of MNA to 4-NA along with concomitant production of HCHO. (•), MNA; (▾), 4-NA; (○), HCHO. (B) Monooxygenation of 4-NA to 4-AP with stoichiometric release of NO_2_^−^. (•), 4-NA; (▾), 4-AP; (○), NO_2_^−^. Values are presented as arithmetic mean of data obtained from experiments carried out in triplicate; error bars represent standard deviation.

### Monooxygenase Activity (Removal of -NO_2_)

The subsequent enzymatic transformation of 4-NA, which was identified as the first metabolite, was also carried out in the above crude cell extract. In the presence of NADPH and FMN cofactor, the crude cell extract showed stoichiometric transformation of 4-NA to 4-AP along with stoichiometric production of NO_2_^−^ (Figure 6B). The specific activity for the conversion of 4-NA to 4-AP was found to be 3.55±0.08 nmol min^−1 ^mg of protein^−1^. No monooxygenase activity was observed in the control reactions that lacked either NADPH or FMN or cell-free protein. The above results showed that the second step of MNA degradation is a flavin-dependent monooxygenation reaction.

### Oxidative Deaminase Activity (Removal of –NH_2_)

The rate of oxygen consumption by 4-AP, 4-chlorophenol (4-CP), and aniline in MNA grown cells of strain FK357 was higher as compared to the MNA and 4-NA (Table 1). However, negligible oxygen consumption was observed by 4-AP, 4-CP and aniline, when 1/4-NB grown cells were incubated with these substrates suggesting the inducible nature of enzyme. In contrast, the lesser amount of oxygen consumption by MNA and 4-NA in 1/4-NB grown cells demonstrated that the pathway enzymes involved in the initiation of MNA degradation have moderate constitutive activities. The inducible nature of enzyme involved in the oxidative deamination of –NH_2_ from aminophenols and anilines are in close agreement with the earlier reports [22], [23], [32], [33]. The stoichiometric release of NH_4_^+^ and formation of BT, chlorocatechol and catechol products from 4-AP, 4-CP and aniline suggested that the deamination of –NH_2_ group is a dioxygenation reaction and also it is inducible in nature.

**Table 1:** Oxygen uptake by MNA-grown and 1/4-NB grown cells^a^.

Substrates	Oxygen uptake (nmol O_2_/min/mg of protein) by cells grown in:	
	MNA	1/4-NB
*N*-Methyl-4-nitroaniline	65.22±0.7	33.19±0.1
4-Nitroaniline	79.50±1.2	28.70±1.1
4-Aminophenol	184.74±0.5	0.27±0.7
4-Chloroaminophenol	173.34±1.3	0.78±0.4
Aniline	190.10±2.1	0.50±0.1

a The reaction was carried in 1.85 ml volume air-saturated phosphate buffer (20 mM, pH 7.2) containing substrates (70 µM), and cells (0.25 mg of protein). Data represents means of at least three separate experiments.

### 1, 2, 4-Benzenetriol 1, 2-dioxygenase Activity

Furthermore, 1, 2, 4-benzenetriol 1, 4-dioxygenase (BtD) activity on BT by crude cell extracts was carried out spectrophotometrically by monitoring time dependent wave length scan over a range of 200–500 nm. During the incubation of BT in crude cell extracts, the substrate peak with proximal absorbance at 283 nm gradually decreased, giving rise to a new peak with maximal absorbance at 243 nm (Figure 7). The absorbance at 243 nm is the characteristic of maleylacetate (MA). The specific activity for the BtD was found to be 2.43±0.30 nmol min^−1 ^mg of protein^−1^.

**Figure 7:** Formation of the maleylacetate (MA) from benzenetriol (BT) by crude cell extracts of *Pseudomonas* sp. strain FK357. Sample and reference cuvette contained phosphate buffer (50 mM, pH 7.0), 10 mM Fe (NH_4_)_2_(SO_4_)_2_.6 H_2_O, and 0.5 mg ml^−1^ protein in a 1.0-ml mixture. The reaction was initiated by addition of 70 µM BT and the spectra were recorded every 1 minute after the addition of BT. The arrows indicate the directions of spectral changes.

## Discussion

Structurally MNA is an analogue to 4-nitroanisole, which contains *O*-methyl group (*O*-CH_3_) and a nitro group (−NO_2_), whereas MNA contains an *N*-methyl group (*N*-CH_3_) and a nitro group (−NO_2_). The mineralization of 4-nitroanisole has been earlier reported by *Rhodococcus* strain AS2 and AS3 [34]. The degradation of 4-nitroanisole starts with *O*-demethylation of *O*-CH_3_ with the formation of 4-nitrophenol, which subsequently get degraded as a result of ring cleavage via the formation of 4-nitrocatechol intermediate [34]. Soil microcosms study demonstrated the possibility of MNA degradation in aerobic conditions. Nitrogen (NH_4_Cl) amended soil microcosms showed the higher rate of MNA degradation as compared to that of unamended soil microcosms. The above result indicates that soil microbes utilizes *N*–CH_3_ group from MNA as the preferential single carbon source i.e. the easiest and first to be used, in the presence of most favourable nitrogen source (NH_4_Cl). Soil microcosms study suggested that microorganisms utilized MNA as sole source of carbon, nitrogen, and energy. Based on the identified intermediates during the growth study, resting cell study and enzyme assays, we proposed a novel MNA degradation pathway in *Pseudomonas* sp. strain FK357 (Figure 8). In this pathway, conversion of MNA into 4-NA is expected to be catalysed by a putative demethylase enzyme capable of removing *N*-CH_3_ via oxidative pathway. *O*-demethylation reactions are widely distributed among microorganisms capable of degrading aromatic compounds containing *O*-CH_3_ group, the removal of *N*-CH_3_ group from aromatic compounds has been shown only in few reports. *Pseudomonas putida* CBB5 has been isolated and characterized for *N*-demethylation reaction occurring in degradation pathway of several purine alkaloids [19], [35]. We were unable to quantify HCHO during the growth study of strain FK357, however, it was later quantified in resting cell study. Enzyme assay carried out for the *N*-demethylation reaction in crude extracts on MNA showed the formation of 4-NA along with stoichiometric production of HCHO. Interestingly, growth yield of strain FK357 on MNA was slightly higher as compared to its growth yield on 4-NA, the possible reason for which could be the availability of extra single carbon source i. e. *N*-CH_3_ from MNA ring. Earlier, it has been reported that the methyl group released either from *N*-methyl or *O*-methyl containing compounds oxidized to HCHO [19], [35], [36], [37], [38], [39], [40], [41]. There are various bacterial strains which have been characterized to utilize HCHO as the sole carbon source [20], [35], [42], [43], [44]. In the presence of nitrogen source, the strain FK357 also utilized HCHO as the sole carbon source (data not shown). Summers et al. [19] characterized *N*-demethylase (Ndm) gene from *Pseudomonas putida* CBB5, which showed the broad substrate activity on several purine alkaloids. Thus, based on the above study, we proposed the involvement of a similar bacterial *N*-demethylation reaction as the first step of MNA degradation. Subsequent degradation of MNA presumably initiated as a result of removal of substituted –NO_2_ or –NH_2_ group from the benzene ring. The mechanism for the removal of –NO_2_ and –NH_2_ groups from benzene ring poses an interesting question and challenge to the microbial systems for the preferential removal of these groups. Usually there are two reaction mechanisms for the removal of –NO_2_ group, one is oxidative and another is reductive [5]. In the oxidative reaction, the removal of –NO_2_ group as nitrite ions (NO_2_^−^) takes place by hydroxylation, while −NO_2_ group get sequentially reduced to nitroso (−NO), hydroxylamine (−NHOH), and amino (−NH_2_) group in the reductive reaction [6], [45], [46]. Another reaction mechanism involves dioxygenation which removes –NO_2_ group by adding two hydroxyl groups simultaneously, one at the nitro-substituted position and the other at the adjacent position [5], [47]. Removal of –NO_2_ group by dioxygenation reaction has been reported earlier in the degradation pathway of nitrobenzene by *Comamonas* sp. strain JS765 [5], [48]. The dioxygenation of –NO_2_ group from nitrobenzene resulted in the formation of 1, 2-*cis*-dihydrodiol product [47], [49]. Similarly, the removal of –NH_2_ group from the benzene ring by dioxygenation reaction has also been reported for the degradation of anilines, diphenylamine, and chloroanilines [22], [23], [32], [50]. Aniline dioxygenase is one of the most commonly characterized enzyme reported for the removal of –NH_2_ group during the aniline and chloroaniline degradation pathways [22], [23], [27], [33], [50], [51].

**Figure 8:** Proposed metabolic pathway for aerobic degradation of MNA by *Pseudomonas* sp. strain FK357.

The crude cell extracts showed conversion of 4-NA into 4-AP with stoichiometric production of NO_2_^−^ and the removal of –NO_2_ from 4-NA occurs via a hydroxylation reaction catalyzed by flavin-dependent monooxygenase (Figure 6A). This reaction is very common for aerobic microbial degradation of nitro or chloro containing aromatic compounds such as 2-chloro-4-nitrophenol, 2-chloro-4-nitroaniline, 4-nitroaniline, 4-nitrophenol, 2, 4-dichlorophenol, and 4-chlorophenol, respectively [6], [21], [33], [52], [53]. Oxygen uptake studies showed the conversion of 4-AP into BT product with stoichiometric release of NH_4_^+^, suggesting that a dioxygenase enzyme catalyses the reaction by introducing two oxygen atoms on the benzene ring. Similar reports has also been shown in case of aniline degradation by strain *Pseudomonas putida* mt-2, *Pseudomonas acidovorans* CA28, *Delftia* sp. AN3, and *Delftia tsuruhatensis* AD9 which degrades aniline via the formation of catechol as the first metabolic product [22], [23], [29], [54]. *Moraxella* sp. strain G is known to mineralize 4-chloroaniline by dioxygenation reaction with the formation of chlorocatechol as a metabolic product along with stoichiometric release of NH_4_^+^ [55]. Furthermore, the crude cell extracts prepared from MNA grown cells also transforms BT to MA, suggesting the involvement of a ring cleavage enzyme i.e. 1, 2, 4- benzenetriol 1, 2-dioxygenase. Formation of MA from BT is commonly reported as a ring cleavage step in 4-nitrophenol degradation pathway [56], [57], [58]. Based on the above identified metabolites, the degradation pathway has been elucidated, showing *N*-demethylation of *N*-CH_3_ group as the first reaction followed by monooxygenase mediated removal of –NO_2_ (Figure 8). Further degradation of 4-AP occurs by the dioxygenation reaction resulting in formation of BT which subsequently gets ring cleaved by 1, 2, 4-benzenetriol 1, 2-dioxygenase enzyme.

## Conclusion

We report isolation and characterization of bacterium *Pseudomonas* sp. strain FK357, which is the first naturally occurring aerobic bacterium capable of utilizing MNA as the sole source of carbon, nitrogen, and energy. Degradation of MNA by strain FK357 occurs via the formation of 4-NA, 4-AP, and BT as major intermediates (Figure 8). Strain FK357 could also be used as an important model system for studies on biochemical and molecular evolution of microbial degradation of MNA. The molecular components involved in the MNA degradation by strain FK357 are yet to be characterized. The future work has been proposed to carry out entire genome sequencing, annotation or genomic library construction of strain FK357 for the characterization of gene(s)/gene cluster involved in this important metabolic pathway.
